RETRACTED

# Detection of Emotion of Speech for RAVDESS Audio Using Hybrid Convolution Neural Network

**DOI:** 10.1155/2022/8472947

**Published:** 2022-02-27

**Authors:** Tanvi Puri, Mukesh Soni, Gaurav Dhiman, Osamah Ibrahim Khalaf, Malik alazzam, Ihtiram Raza Khan

**Affiliations:** ^1^ICT Ganpat University, Ahmedabad, Gujarat, India; ^2^Computer Science and Engineering, Jagran Lakecity University, Bhopal, India; ^3^Department of Computer Science, Government Bikram College of Commerce, Patiala, India; ^4^University Centre for Research and Development, Department of Computer Science and Engineering, Chandigarh University, Gharuan, Mohali, India; ^5^Department of Computer Science and Engineering, Graphic Era Deemed to be University, Dehradun, India; ^6^Al-Nahrain University, Baghdad, Iraq; ^7^Lone Star College-Victory Center, Houston, TX, USA; ^8^Computer Science Department, Jamia Hamdard University, Delhi, India

## Abstract

Every human being has emotion for every item related to them. For every customer, their emotion can help the customer representative to understand their requirement. So, speech emotion recognition plays an important role in the interaction between humans. Now, the intelligent system can help to improve the performance for which we design the convolution neural network (CNN) based network that can classify emotions in different categories like positive, negative, or more specific. In this paper, we use the Ryerson Audio-Visual Database of Emotional Speech and Song (RAVDESS) audio records. The Log Mel Spectrogram and Mel-Frequency Cepstral Coefficients (MFCCs) were used to feature the raw audio file. These properties were used in the classification of emotions using techniques, such as Long Short-Term Memory (LSTM), CNNs, Hidden Markov models (HMMs), and Deep Neural Networks (DNNs). For this paper, we have divided the emotions into three sections for males and females. In the first section, we divide the emotion into two classes as positive. In the second section, we divide the emotion into three classes such as positive, negative, and neutral. In the third section, we divide the emotions into 8 different classes such as happy, sad, angry, fearful, surprise, disgust expressions, calm, and fearful emotions. For these three sections, we proposed the model which contains the eight consecutive layers of the 2D convolution neural method. The purposed model gives the better-performed categories to other previously given models. Now, we can identify the emotion of the consumer in better ways.

## 1. Introduction

Speech is the direct way to transfer information from one end to another end. It contains a wide variety of information, and it can express rich emotional information through the emotions it contains and visualize it in response to objects, scenes, or events. The automatic recognition of emotions by analyzing the human voice and facial expressions has become this subject. The following systems can be cited as an example of the areas in which these studies are used and their intended use is provided:

- Education: A course system for distance education can detect bored users so that they can change the style or level of the material provided and, in addition, provide emotional incentives or compromises.
- Automobile: Driving performance and the emotional state of the driver are often linked internally. Therefore, these systems can be used to promote the driving experience and to improve driving performance.
- Security: They can be used as support systems in public spaces by detecting extreme feelings such as fear and anxiety.
- Communication: In call centers, when the automatic emotion recognition system is integrated with the interactive voice response system, it can help improve customer service.
- Health: It can be beneficial for people with autism who can use portable devices to understand their feelings and emotions and possibly adjust their social behavior accordingly [1].

RETRACTED

It is known that some physiological changes occur in the body due to people's emotional state. Some variables such as pulse, blood pressure, facial expressions, body movements, brain waves, and acoustic properties vary depending on the emotional state, pulse, blood pressure, brainwaves, and so forth. Although changes cannot be detected without a portable medical device, facial expressions and voice signals can be received directly without connecting any device to the person. For this reason, most studies on this topic have focused on the automatic recognition of emotions using visual and auditory signals. However, acoustic signals are the most used data after facial signs to identify a person's emotional state [2].

Many solutions, mechanisms, and methods for the identification of feelings from expression have been suggested. Some elements of such works are nevertheless also marginalized:

- Often, it is an unambiguous job to delineate emotion: angry people can talk in a noisy, high-pitched voice, but another person can convey rage with a silent and stronger voice. It also varies according to the mood and attitude of an individual, but no device can accurately evaluate the sentiment of an individual based on those features of their expression.
- A large portion of SER studies neglects data mismatch (speech emotional recognition). If one emotion has more data than any other emotion to balance it, the model(s) conquer the emotion and struggle to distinguish the others accurately.

RETRACTED

While the overall consistency of the designation can be seen, the paradigm in truth cannot be used as a diverse emotional recognition system that can identify a spectrum of emotions. There must also be resampling and optimization strategies used when developing SER structures (that is to say if the databases involved are imbalanced). In the case of such imbalances, precision as the required assessment metric is often ambiguous and precise. Unfortunately, the primary assessment was consistency taking into account these considerations; research into speech emotion detection has been loosely split into two parts: speech-independent and speech-independent. We address the latest trends both following a historical review of proposals suggested. Besides, a more detailed SER study analysis can be found in [3–6].

The above systems are some of the most common in the region of SER. Any other emotionally accepted machine-learning models are as follows:

- K Nearest Neighbors: Classification systems that assign a particular sample to the “nearest neighbor“ mark. Different distance considerations like Euclidean distance, Manhattan, cosine similarity measure, Minkowsky, correlation, Chi-square, etc. can be used for the nearest neighbor criteria. K is essential to the classifier's efficiency. On the SER KNN classifiers, there is not much literature; there are some in [1, 7].
- Trees: Trees are nonparametric learning activities that learn inference rules, patterns, and samples from their underlying data. Many implementations of the decision tree are included, such as CART, C4.5, CHAID, QUEST, ID3, and J48. Decision trees are used also for ensemble methods like random forests or boosted trees as simple estimators. Any SER studies can be found at [2, 8, 9] on the use of trees.
- Ensemble: Ensemble learning blends several machine-learning models to increase efficiency. Several assembly methods can be classed loosened into bagging (aggregation of bootstraps), boosting, or voting (a generalization of stacked systems). Some works discuss these various SER classifiers in [10, 11].

The following identifies some of the key forms of neural networks behind profound learning systems.

- Deep Neural Network (DNN): DNN is an artificial neural network (ANN), with many hidden layers.“deep“ denotes a large number of these layers. The depth permits learning representations and critical characteristics to be categorized. DNNs in a wide range of areas have been widely used and they are essential in SER.
- Convolution Neural Network (CNN): Convolution Neural Network (CNN) is an extension of DNN that operates on data that come in the form of several arrays, in particular images. Much as with signals represented as a single-dimensional array, the input has philters that are screwed over it and then packed together for a smaller dimension. This is done to collect local input data, and if replicated, a hierarchy of features is created.
- Long Short-Term Memory (LSTM): It is a modified version of a recurrent neural network which overcomes the vanishing gradient problem. RNNs hold a vector of the state that includes details on all previous elements' chronological history. The gradients measured during RNN preparation, however, are explosive or disappear very rapidly over several time stages, leading to inadequate capture of long-term dependence. Therefore, long-term memory (LSTM) networks with three special gates named input gate, forget gate, and output gate are used to manage long dependencies without underflow or overload.
- Autoencoders: Autoencoders are particular types of unmonitored DNNs that are used first to recreate and then reconstruct the input to a latent spatial representation (encoding). This structure will also be used not only to Denise but also to decrease dimensionality.
- Warning: The principle of concentration, focused loosely on how people focus on a specific portion of the input at high resolution and all other sections with lower resolution, is an improvement to the above approaches. The attention mechanism helps one to “respect“ only the appropriate input pieces at each point of the output generation. Diverse networks, their architectures, and their functions are defined in detail in [12].

RETRACTED

The paper is organized as follows.  Section 2 presents the literature review of the recognition of speech emotions.  Section 3 describes the methods of our proposed system. In Section 4, the experimental results are presented. And finally, in Section 5, we conclude our work.

### 1.1. Literature Review

In recent years, neural network architectures and end-to-end systems in many areas have seen a tremendous upsurge. Deep learning has been one of the most commonly used learning approaches for problems from speech acknowledgment to operating cars. The success of profound learning solutions for many problematic areas can be due to this model systems' willingness to carry out practical learning alone, rather than to attempts for handcrafted functionality.

Out of these, DNNs [2] and DCNNs [13], more profound than CNN, were the first two deep-learning approaches. The roles of the profound learning techniques in the field of the automated recognition of speech [14], the imagery classifying [13], and object detection [15] were played automatically by learning feature representations from raw input data.

RETRACTED

It is therefore a fair step to examine SER approaches to deep learning. For example, in the classification of emotion, the neural network [14] was used to learn high-level characteristics from the low-level traits derived at an acoustic level. DNNs were some of the first ones to be tested. But the previous study did not take due account of proper elimination of the feature, so the findings were typically unfaithful.

In this first study [16], a DNN carries on the features collected at the acoustic level and generates a distribution of the likelihood on the segmental emotional level. The attributes are used to assess the emotional class. An extreme learning machine (ELM) [17] is the addition of a neural network with one hidden layer which is used to conduct a classification of emotional characteristics on the utterance level. During training, ELM does not require weight replication. An ELM network is not needed for a large quantity of training data because the segment-level output already provides a significant amount.

Later works [18] used CNNs in the case of speech signals for the learning of functionality. Mao et al. [19] suggested a strategy for the learning of CNN effectiveness by CNN in the form of the fact that in CNN basic features are learned in the lower layers. Their analysis has demonstrated the two-phase CNN learning concept. In the first step, the data is based on data that are not known to learn local characteristics which are invariant with the aid of a sparse autoencoder and in the second phase the use of SDFA as an extractor for characteristics to learn discriminative characteristics that impact the input to SDFA. This was the first thesis to propose functional learning to SER and illustrate how CNNs can be modeled successfully to extract an optimized functional package.

Trigeorgis et al. [20] proposed a two-layer CNN-based end-to-end SER with a long short-stack (LSTM) network. Bhargava and Rose [21] also noted that deep networking's intermediate representations do not vary significantly from the talk-making functions. In contrast to the Log Melfilterbank energy, Sainath et al. [22] suggested a convolutional LSTM-DNN, demonstrating that speech signals are best temporarily and contextually modeled by their systems. The aforementioned explanations are the use of the pipeline end to end and, thus, characteristics are accomplished by convolutions, and LSTMs are employed to set a standard ground with reference to other architectures suggested in contexts.

Another research suggesting the use of LSTM CNNs for SER is [23]. So far, most strategies have concentrated on extracting a decent number of features and feeding them to a dense rank. The emphasis on recording variance of features over time has been very small. The EmNet function introduced in [23] uses not only a default feature collection but also feeds into a CNN feature that removes local dependencies and then modes higher-level functions using a worldwide convolution layer. Finally, this layer's output is passed to an LSTM network, so a variety of features are applied to this thick network.

RETRACTED

Emphasis on Time convolutions/1D Frequency [18, 19] instead of 2D or 3D convolution used in the DCNN models [13] is important to notice that the above-mentioned architectures concentrate. They are also simplistic models, i.e., one or two layers of CNNs were used, while the DCNN models were even more profound. Later investigations found that in the field of vision deep multilevel networks composed of convolutional and pooling layers were greater than those of CNNs [22, 23]. That the DCNN will maintain the hierarchical existence of the knowledge is the explanation behind that observation.

To build an efficient method for emotional identification, the emphasis is on the performance of models of greater depth [24]. Three Log Mel spectrograms from one-dimensional utterances were used for the methodology suggested in this project [25]. There were also suggestions for integrating time-limit matching with optimum Lp-norm bundling to gain utterance-level characteristics from segment-level characteristics.

In all the works listed above, no account has been taken of the fact that a DNN uses custom features as feedback. Consequently, the models constructed cannot be generalized enough, since particular functions are influenced by multiple parameters such as expression and material. We may describe individual features as numerical values that are specifically expressed in the personal details that do not represent an invariable quantity. Therefore, because of personal characteristics reliance, SER achieves positive results in the study of the speaker-dependent.

Because of the good performance of Mel-frequency cepstral coefficients (MFCCs) in emotional recognizing systems with deltas and double delta functions [25], it is possible to say that measured deltas and delta deltas can represent emotional transition and retain emotional information while minimizing the effect of not very significant features. Another case in point is [24] that reveals the input to the coevolution recurrent network of deltas and double deltas. In contrast to their baseline, the DNN–ELM model [16], Cheng et al. [25] evaluated carefully layered RNNs registered an improvement of 11.26 in Emo-DB and 111.26%, in IEMOCAP.

Rasmus et al. [26] developed the idea of pure unattended networks that conserve adequate information, in comparison with strictly supervised networks, to recreate input instances that only hold specific classification information. This kind of architecture assumes that all of these features are a semisupervised ladder network architecture. According to studies in speech context [27], a denoising autoencoder (DAE) is used to insert noise into all hidden layers and link the noisy encoder and decoder pair with the Skip links. The output of the encoder functions as the SVM function. Cross-entropy costs of the encoders with the expense of restoration by the decoders constitute the loss function.

RETRACTED

## 2. Materials and Methods

### 2.1. Data Description

The RAVDESS [28] dataset was picked as it consists of speech and song records, categorized into eight separate levels by 247 untrained Americans: Relaxed, Happy, Sad, Furious, Afraid, Disgust, and Surprise and a neutral base for each performer. The following table offers a breakdown of the emotional groups in the dataset shown in Figure 1.

- The data collection consists of 24 trained performers, 12 males and 12 females. Gender-balanced.
- In a standardized setting, the audio files were generated and each contains the same statements in an American focus. There are also two related file types:
- The speech file contains 1440 files: 60 trials per actor x 24 actors = 1440 speech files (audio speech actor 01–24.zip, 215 MB).
- The audio file includes 1012 files (audio song actors 01–24.zip, 198 MB): 44 actor evaluations x 23 actors = 1012.
- Both types of audio files have the 16-bit bitrate and 48 kHz sampling rate in the WAV raw audio file format. Both recordings are uncommented, lossless audio, ensuring that no data/information is missing or changed from the initial recording of the audio files in the dataset.

As mentioned earlier, we used the libROSA python package to process/manipulate these scripts. This kit was designed to be the best collection for our dataset for music and audio research.

We read in one WAV file at a time after importing libROSA. A 1-dimensional array-specific audio time series with a stereo time sample rate (which determines the array length) where the elements inside each array reflect the sound wave amplitude is given by the libROSA 'load' function. The output is shown in Figure 2.

### 2.2. Data Preprocessing and Exploration

We will clarify some of the principles that allow us to pick our characteristics before moving into preprocessing and data exploration.

 
**Mel scale**: a scale of pitches judged by listeners to equate with each other's sense of frequency.
 
**Pitch**: the pitch or the level of sound. It depends on the frequency, the higher the frequency is.
 
**Frequency**: vibration rate for sound, wave cycles measurements per second.
 
**Chroma**: audio representation where spectrum is projected on twelve bins containing twelve different semidimensions. Computed by applying the spectrum of log frequency to octaves.
 
**Fourier Transforms**: used for moving to the frequency domain from the time domain. Time domain displays the changes in the signal over time. The frequency domain indicates that a spectrum of frequencies contains a variety of signals within the frequency band.

RETRACTED

The following functions were used to derive MFCC, Chroma, and Mel spectrograms from the raw audio file and some of the functionalities of libROSA's audio processing.

The filename (path) will be obtained and the audio file will be loaded using the libROSA library. Many libROSA functions are used for removing functionalities which are then aggregated and returned as a NumPy list.

Proposed Model: we have proposed a model which you can see in Figure 3. It shows that this model uses the ReLu function for the activation to the model to overcome the problem of vanishing of the gradient for that we also do the batch normalization two times: first was the initial layer of the CNN and the second was the center of the model.

Proposed Algorithm: in Figure 4, we show our stop that was used to develop the algorithm.

## 3. Results and Discussion

For the computation of these results, we use the Google collab for running the code. First, we perform the distribution of the data in equal formate. We visualize the audio file as waveform and its spectrogram as shown in Figure 5. Then, we find out that the initial and the end one second is not having any kind of autosignal in the waveform. So, for all the audio files, we remove this one and last second from the audio file.

MFCC, Chroma, and Mel spectrograms from the raw audio file which show the different patterns for the different types of emotion are shown in Figure 6 which we are trying to recognize correctly.

We prepare our model using CNN which executes the 700 epoch in the batch of 32; now, in the given Figures 7(a) and 7(b), our model accuracy is more than 98% which is better than any of the other models.

## 4. Conclusion and Discussion

The modern age of automation is characterized by the emerging growth and advancement of artificial intelligence and machine learning. Many automatic systems function using the user's voice recognition. There can be several benefits over current systems if the computers can recognize the mood of the speaker (user) in addition to understanding words. The need for a speech emotion recognition system involves electronic call-center calls, computer-based training applications, a care diagnostics tool, and an automatic translation system.

RETRACTED

This theory suggested a new profound learning paradigm to receive sound and to derive voice signals, such as MFCCs, short-term energy, and spectrogram entropy coefficients. The functions that are focused on the changes in the audio timing reflect details on the speaker's changes in audio and minimize customized speaking features of the speaker. Although the suggested approach of audio depression recognition using a convolution network has produced reasonable outcomes, the choice of speech segments has a significant impact on the final results.

This study explored in depth the steps to construct a framework of speech emotional detection and performed multiple experiments to explain the effect of each point. The small number of public speaker databases initially made it impossible for a well-educated model to be adopted. Next, many new methods were suggested in earlier studies to obtain characteristics, and several studies were carried out to find the best method. Finally, the selection of classification required learning about the intensity and vulnerability of each emotion detection classification algorithm [29, 30]. At the end of the trial, an interconnected feature space can be concluded to deliver a higher recognition rate than a single feature [29–32].

## Figures and Tables

**Figure 1:** RAVDESS dataset.

**Figure 2:** Distribution of data RAVDESS dataset.

**Figure 3:** Proposed model for the SER.

**Figure 4:** Proposed algorithm.

**Figure 5:** The audio file's waveform and its spectrogram.

**Figure 6:** Mel power spectrogram.

**Figure 7:** (a) Plotting the Train Valid Loss Graph. (b) Actual v/s predicted emotions.

## Data Availability

The data used to support the findings of this study are available from the author upon request (mukesh.research24@gmail.com).
